The article "Dieckol inhibits non‐small–cell lung cancer cell proliferation and migration by regulating the PI3K/AKT signaling pathway" was retracted in 2026. Reasons: plagiarized images; content taken from a thesis; overlap with other authors' work; unreliable results or conclusions.

# Dieckol inhibits non‐small–cell lung cancer cell proliferation and migration by regulating the PI3K/AKT signaling pathway

**DOI:** 10.1002/jbt.22346

**Published:** 2019-07-10

**Authors:** Chun‐Hong Wang, Xiao‐Feng Li, Li‐Fang Jin, Yan Zhao, Geng‐Jun Zhu, Wei‐Zhang Shen

**Affiliations:** ^1^ Department of Oncology and Hematology The Second Hospital of Jilin University Changchun Jilin China

**Keywords:** anticancer drug, cadherin, dieckol, lung cancer, NSCLC, PI3K/AKT/mTOR

## Abstract

Non‐small–cell lung cancer (NSCLC) is one of the most prevalent type of lung cancers with an increased mortality rate in both developed and developing countries worldwide. Dieckol is one such polyphenolic drug extracted from brown algae which has proven antioxidant and anti‐inflammatory properties. In the present study, we evaluated the anticancer property of dieckol against NSCLC cell line A549. The LC_50_ value of dieckol was found to be 25 µg/mL by performing 3‐(4,5‐dimethylthiazol‐2‐yl)‐2,5‐diphenyltetrazolium bromide (MTT) assay and the antiapoptotic property of dieckol was analyzed by dual staining technique with acridine orange/propidium iodide (AO/PI) stains. It was further confirmed with flow cytometry analysis with Annexin FITC and JC‐1 staining and the anti‐invasive property was assessed by Transwell assay. The molecular mechanism of dieckol anticancer activity was confirmed by estimating the levels of caspases and by estimating the signaling proteins of Pi3K/AKT/mTOR signaling pathway using the immunoblotting technique. Our data suggest that dieckol is potent anticancer agent, it effectively inhibits the invasive and migratory property A549 cells and it also induces apoptosis via inhibiting Pi3K/AKT/mTOR signaling, activating the tumor suppressor protein E‐cadherin signifying that dieckol is potent natural anticancer drug to treat NSCLC.

## 1 INTRODUCTION

Cancer is one of the prevailing cause of death in both developed and developing countries worldwide. It has been estimated at the year of 2027 there will be 70% increase in the rate of cancer‐related deaths. Among all cancer types about 45% of cancer, deaths are due to the prevalent cancers like lung, prostate, breast, and colorecturm.^1^ Lung cancer is one of the most widespread cancer which accounts for about 30% of cancer‐related death.^2^, ^3^ In India, the survival rate of patients with lung cancer is only about 17.8% and the highest incidence of lung cancer was reported in Mizoram.^4^ Lung cancer has been classified into non‐small–cell lung cancer (NSCLC) and small‐cell lung cancer (SCLC) depending upon their invasive property.^5^ SCLC is malignant tumor which accounts for about 15% of lung cancer remaining 85% are contributed by the NSCLC. NSCLC were further divided to adenocarcinoma (38.5%), squamous cell carcinoma (20%) and large cell carcinoma (3.5%).^6^

PI3K/AKT/mTOR signaling regulates cell proliferation, differentiation, cellular metabolism, and cytoskeletal reorganization leading to apoptosis and cancer cell survival. Activation of the PI3K/AKT/mTOR signaling pathway mediated through molecular aberrations in promoting tumor development as well as resistance to anticancer therapies.^7^ PI3K/AKT/mTOR signaling pathway is one of the most recurrently deregulated pathway in all cancer condition especially it is reported in NSCLC.^8^ Fifty percent to seventy percent of NSCLC patients were reported with increased expression of phosphorylated AKT protein which continuously activates the downstream molecules of PI3K/AKT/mTOR signaling pathway.^9^, ^10^ The strict regulation of tumor suppressor protein also plays a key role in cancer progression, one such protein is E‐cadherin. E‐cadherin regulates the epithelial to mesenchymal transition of cells which is one of the key events in cancer cell progression.^11^, ^12^, ^13^

Recently research on targeted cancer therapy is been evolving and most of the researchers are investigating the potential of herbal drugs to inhibit the deregulated PI3K/AKT/mTOR signaling pathway. Since NSCLC were mostly diagnosed at the advanced stages, the survival rate of patients is much less.^14^ Alone or combinations of chemotherapy, radiotherapy, and surgery are the only options for NSCLC patients, but they are less potent and they induce severe side effects.^15^ Therefore treating NSCLC patients with the potent herbal based drug with less or nil side effects are the need of today.

One such drug is dieckol, a polyphenolic compound found in brown algae *Ecklonia cava*.^16^ Dieckol possesses multifunctional pharmacological activities such as antioxidant, antiaging, antiallergic, antihyperlipidemic, anti‐inflammatory, antidiabetic, antitumor and antineurodegenerative.^17^, ^18^ Moreover, DEK inhibits human breast carcinoma, liver, and ovarian cancer cell proliferation.^19^, ^20^, ^21^ Even though it has been reported to possess anticancer activity the molecular mechanism of its anticancer property yet not elucidated. Hence the present study is designed to detect the anticancer effect of dieckol against the NSCLC cells A549. Before analyzing the anticancer potential of dieckol we proposed to analyze the cytotoxic effect, cell invasion, migration, and apoptotic induction in A549 cell line. To confirm the induction of apoptosis by dieckol we analyzed the PI3K/AKT and apoptotic signaling molecules in dieckol treated A549 cells.

## 2 MATERIALS AND METHODS

### 2.1 Materials

Dieckol (AKOS032954113) was purchased from AKos Consulting & Solutions, Culture medium Dulbecco's modified Eagle's medium (DMEM), fetal bovine serum (FBS), and antibiotics were purchased from Gibco. Antibodies were purchased from Santa Cruz Biotechnology, Inc. All other chemicals used were superior quality purchased from Sigma chemicals.

### 2.2 Cell culture

A549, human NSCLC cell lines were purchased from the Institute of Biochemistry and Cell Biology, Chinese Academy of Sciences (Shanghai, China). Cells were cultured in DMEM, the medium was supplemented with 10% FBS, and 1% of antibiotic/antimycotic solution penicillin and streptomycin at 37°C with 5% CO_2_. Upon reaching 80% confluency the cells were trypsinized with 0.25% trypsin and 0.02% ethyldiaminetetaacetic acid (EDTA) for further subculturing. The cell lines were treated with different concentrations of dieckol (5, 10, 25, 50, 75, and 100 µg/mL) dissolved in dimethyl sulfoxide (DMSO) as that the final concentration of DMSO in the medium was 0.1%.

### 2.3 Cytotoxicity assay of dieckol in lung cancer cells

The cells were counted and approximately about 5 × 10^3^ cells were plated in 96‐well plate and incubated for 24 hours at temperature of 37°C. After 24 hours the culture medium was replaced with culture medium containing different concentrations of dieckol (5, 10, 25, 50, 75, 100 µg/mL), control wells were treated with plain medium. After incubation, to each well 20 µL of 3‐(4,5‐dimethylthiazol‐2‐yl)‐2,5‐diphenyltetrazolium bromide (MTT) was added and incubated for 4 hours at 37°C. The formazan crystals formed by the reduction of MTT by mitochondrial succinic dehydrogenase secreted by viable cells were dissolved using 150 µL of DMSO. The absorbance was measured at 450 nm and the LC_50_ value of dieckol was calculated.

### 2.4 Acridine orange/propidium iodide dual Staining of dieckol in lung cancer cells

The induction of apoptosis by dieckol on A549 cell line was assessed by dual staining technique. Acridine orange (AO) stains all the cells irrespective of dead or alive whereas the propidium iodide (PI) stains only the dead cells, thus the induction of apoptosis by dieckol can be easily assessed. The treated cells were fixed using 0.1% of Triton X‐100 and then stained with 0.67 µM of acridine orange and 75 µM of PI for 15 minutes, viewed under fluorescent microscope. The alive cells fluoresce in green color whereas the dead cells fluoresce in red color.

### 2.5 Flow cytometry analysis of dieckol in lung cancer cells

The induction of apoptosis by dieckol on A549 cell line was assessed by flow cytometry after staining with Annexin V‐fluorescein isothiocyanate (apoptosis detection kit) and propidium iodide. The treated cells were centrifuged at 800*g* for 5 min at 4°C and the pellet was collected, washed with precooled phosphate‐buffered solution (PBS) and again centrifuged. The pellet was resuspended with PBS and 10 µL of Annexin V‐FITC was added and incubated for 15 minutes at dark. After incubation, the cells were stained with 5 µL propidium iodide for 5 minutes. The cells were then assessed with fluorescence‐activated cell sorter (FACScan, BD) to detect the apoptotic and necrotic cells. The mitochondrial membrane disruption of the cells was assessed by staining with JC‐1 stain.

### 2.6 Wound‐healing assay of dieckol in lung cancer cells

The inhibitory potential of dieckol toward cell migration of A549 cell line was assessed by wound‐healing assay. A549 cells were plated in six‐well plates and incubated for 24 hours at 37°C with 5% CO_2._ After 24 hours, upon obtaining 90% confluency the cell were starved for 6 hours and an artificial wound was created by scratching the cell monolayer with 10 μL micropipette tip. The floating cells were washed twice with PBS and the plates were replaced with serum‐free DMEM medium along with dieckol (25 and 50 µg/mL concentrations), incubated with 5% CO_2_ for 24 hours at 37°C_._ The migration of cells from the scratched edges was photographed using phase‐contrast microscope at 0 and 24 hours. The wound closure rate was calculated using the formula:

$$\frac{\text{Initial width}\;@\;0h-\text{Final}\;\text{incision}\;\text{width}\;@\;\text{24h}\;\times \text{100}}{\text{Initial width}\;@\;0h}.$$

### 2.7 Transwell‐invasion assay of dieckol in lung cancer cells

Effect of dieckol on inhibiting the invasive property of A549 lung carcinoma cells were analyzed by performing matrigel invasion assay. Before suspending in serum free DMEM medium with dieckol (25 and 50 µL/mL) and without dieckol as control, the trypsinized A549 cells were rinsed with PBS. 0.2 mL containing about 10^5^ cells was seeded in the upper chamber of Transwell inserts coated with Matrigel (Becton Dickinson). The lower chamber is filled with 0.4 mL DMEM/F12 medium with 10% FBS (act as chemoattractant) and incubated for 24 hours. After 24 hours the migrated and adherent cells on the upper and lower surface, respectively, were stained with Diff‐Quick stain and viewed using fluorescence microscopy (NIKON Eclipse 80i, Japan).

### 2.8 Caspases activity of dieckol in lung cancer cells

Caspases are the key factors which initiate and execute apoptosis; the ability of dieckol to activate caspases was assessed by caspase activity assay. The activity of proteases caspases were detected using the caspase‐3 (ab39401), caspase‐8 (ab39700), and caspase‐9 (ab65608) kits purchased from Abcam. The caspases‐3, ‐8, and ‐9 recognizes the sequence DEVD, IETD, and LEHD, respectively, and cleaves from the labeled substrate p‐NA emitting light which was quantified using spectrophotometer at 400 to 405 nm.

### 2.9 Immunoblotting analysis of dieckol in lung cancer cells

When the cell reaches the confluence of 80%, the cells were treated with dieckol (25 and 50 µL concentrations) and the control cells were treated with 0.1% DMSO, incubated for 24 hours. After 24 hours incubations the cells were lysed with radioimmunoprecipitation assay (RIPA) buffer and the protein concentration was measured using Bradford reagent. Fifty micrograms of total protein from each group were heated at 95°C for 5 minutes and then electrophoresed using 10% sodium dodecyl sulfate polyacrylamide gel electrophoresis. The separated protein were transferred to polyvinylidene difluoride (PVDF) membrane and then the membrane were blocked with 5% skimmed milk for 1 hour at room temperature. After blocking the membrane were washed and incubated with primary antibodies E‐cadherin, (sc‐7870), N‐cadherin (sc‐59987), vimetin (sc‐24613), Twist (sc‐170453), MMP9 (sc‐21733), uPA (sc‐59727), P‐PI3K (sc‐4228), PI3K (sc‐1637), P‐AKT (sc‐7985‐R), AKT (sc‐5298), P‐mTOR (sc‐101738), mTOR (sc‐1549), p70S6K (sc‐230), cyclin D1(sc‐753), actin (sc‐1616) for overnight at 4°C. The membranes were washed after incubation and then incubated with secondary antibodies for 1 hour at room temperature. After incubation, the membranes were washed and the bands were visualized using chemiluminescence reagent (PerkinElmer, Inc) and the bands were quantified using Quantity One Software (Bio‐Rad)

### 2.10 Statistical analysis

The obtained data were statistically analyzed using GraphPad prism software (Graph Pad Software, Inc, San Diego, CA) and expressed as mean ± standard deviation. One way analysis of variance followed by SNK post hoc test was performed to analyze the significant difference between the groups. *P* values were considered as *P* < .05

## 3 RESULTS

### 3.1 Effect of dieckol on A549 cell viability

To assess the effect of dieckol on A549 cell viability MTT assay was performed. Compared with the control there is constant decrease in the cell viability with regard to increased concentration of dieckol treatment. Only 50% of cells were alive in cells treated with 25 µg/mL dieckol, therefore for the further studies, the dosage 25 and 50 µg/mL were selected (Figure 1A).

**Figure 1:** Cytotoxic effect of dieckol against non‐small–cell lung carcinoma A549 cell line. A, Each bar represents mean ± SEM of three independent observations. *P* < .05 is considered as statistically significant. B, Increased number of apoptotic cells with membrane blebbing, DNA fragmentation and chromatin condensation were observed in 50 µg/mL diekol treated group and positive control. *P* < .05 is considered as statistically significant

### 3.2 Apoptotic effect of dieckol on A549 cell line

The induction of apoptosis by dieckol on A549 cell line was assessed by AO/PI dual staining technique. The A549 cells treated with 25 µg/mL dieckol (Figure 1B) showed lesser number of apoptotic cells with blebbed nucleus, fragmented DNA, condensed chromatin compared with 50 µg/mL dieckol and positive control (Figure 1B). Fifty micrograms per milliliters dieckol treated cells showed few number of necrotic cells which are with diffused chromatin and apparently disrupted nuclear membrane (Figure 1B).

To confirm the anitapoptotic effect of dieckol, the A549 cells treated with different concentration of dieckol were subjected to flow cytometry analysis. Twenty‐five micrograms per milliliters dieckol treated cells showed 79.34% of viable cells whereas it is further decreased to 51.77% in 50 µg/mL dieckol treated group. Compared with control the early apoptotic and late apoptotic cells were increased respectively in 25 (8.04% and 10.33%) and 50 µg/mL (21.74% and 22.66) dieckol treated groups (Figure 2). There is no much difference was observed in necrotic cell populations in control and treated groups. Further the mitochondrial membrane potential (MMP) disruption in cells by dieckol was estimated by staining the cells with JC‐1 stain and subjecting it to flow cytometry analysis. Increased percentage of MMP disruption was observed in 50 µg/mL (16.52%), 25 µg/mL (12.98%), whereas it is only 3.6% in control group (Figure 3).

**Figure 2:** Flow cytometric analysis in A549 cells for 24 hours using the Annexin V/FITC and mitochondrial membrane potential with dieckol of various concentrations. Each bar represents mean ± SEM of three independent observations. *P* < .05 is considered as statistically significant. FITC, fluorescein isothiocyanate

**Figure 3:** Effect of dieckol on cell invasion and migration in non‐small–cell lung carcinoma A549 cell line. Each bar represents mean ± SEM of three independent observations. Representative images were shown at the magnification of ×100. The wound closure rate (A) and percentage of cell invaded (B) were calculated and represented as bar diagram. Each bar represents mean ± SEM of three independent observations. *P* < .05 is considered as statistically significant

### 3.3 Dieckol inhibitory property against A549 cell invasion

Transwell assay was performed to assess the effect of dieckol on A549 carcinoma cell line invasion and migration, which are the hallmarks of cancer progression. Dieckol exhibited significant inhibition of both cell invasion and migration property of A549 (Figure 3), when compared with 25 µg/mL concentration of dieckol treatment, in 50 µg/mL treated group the cell invasion and migration were decreased to 50% and 70%, respectively.

### 3.4 Effect of dieckol on caspases

Caspases are the cysteine‐aspartate proteases which play an important role in apoptosis. Caspases‐3 are the initiator caspases and caspase‐8, caspase‐9 are executor caspases. Both the initiator and the executor caspases were increased in NSCLC cells A549 treated with 25 and 50 µg/mL of dieckol (Figure 4). Compared with control the caspases activities were increased, respectively, by 20% and 35% in 25 and 50 µg/mL of dieckol treated cells.

**Figure 4:** Effect of dieckol on caspases non‐small–cell lung carcinoma A549 cell line. The activation of caspases by dieckol treatment were quantified and their activity were represented as bar diagram for caspase‐3 (A), caspase‐8 (B), and caspase‐9 (C) Each bar represents mean ± SEM of three independent observations. *P *< .05 is considered as statistically significant

### 3.5 Dieckol effect on cell adhesion proteins

The cell‐cell adhesion, tissue homeostasis were regulated by cadherin‐catenin proteins. E‐cadherin, N‐cadherin and its downstream molecules play a major role in cell proliferation and migration of tumor cells. In the present study, the cells treated with 25 and 50 µg/mL dieckol showed increased expression of E‐cadherin protein and subsequently decreased expression of N‐cadherin, structural protein vimentin, Twist, matrix metalloproteinases‐9 (MMP9), and uPA (Figure 5A).

**Figure 5:** Immunoblotting analysis of E‐cadherin & PI3K/AKT signaling proteins. Effect of dieckol on cell adhesion signaling molecules in non‐small–cell lung carcinoma A549 cell line. Each bar represents mean ± SEM of three independent observations. *P *< .05 is considered as statistically significant

### 3.6 Inhibitory effect of dieckol on PI3K/AKT signaling pathway in A549 cell line

PI3K/AKT signaling is a key signaling pathway involved in cell proliferation and migration. Significant increase in PI3K/AKT signaling was observed in most of the cancer condition. Since in our present study dieckol potential inhibited the cell invasion and migration, we assessed the molecular mechanism involved by evaluating the levels of PI3K/AKT signaling molecules after dieckol treatment. Increased expression of PI3K and its downstream molecules AKT, mTOR, p70S6K, and cyclin D1 (Figure 5B) were observed in control group whereas it is significantly decreased in 25 and 50 µg/mL dieckol treated groups.

## 4 DISCUSSION

Dieckol is polyphenolic compound isolated from *E. cava* brown algae consumed by the people of Asia and Europe.^22^ It belongs to the family of Lessoniaceae and it also used as in Japan and Korea.^23^ The major components present in *E. cava* are phlorotannins and flucoidans which posses various biological properties. Phlorotannins are unique polyphenolic compounds which are produced by the polymerization of phloroglucinol. Phloroglucinol possess different chemical structure compared with terrestrial plant polyphenols. There are different types of pholorotannins namely eckol, dieckol, triphlorethol‐A etc.^24^, ^25^, ^26^ Dieckol possess antioxidant, anti‐inflammatory, anitidabetic, antibacterial activity.^27^, ^28^, ^29^ In the present study, we assessed the anticancer property of dieckol against the NSCLC cell line A549, which is most prevalent type of lung cancer and the survival rate is also poor.

Cytotoxicity assay was performed with different concentrations of dieckol (5‐100 µg/mL) to assess effective IC_50_ dose dieckol against A549 cell line. The most effective inhibition of A549 cells was observed at the dose of 100 µg/mL and IC_50_ was obtained at the dose of 25 µg/mL concentration. Hence for the further studies to assess the anticancer activity of dieckol the dosage of 25 and 50 µg/mL were selected. The apoptotic activity of dieckol against A549 was assessed by dual staining technique with AO/PI nuclear stain. AO stain which imparts green colour fluorescence is permeable to both the live and dead cells whereas the PI which stains the nucleus in red colour is permeable only to the dead cells. Compared with control the 25 µg/mL and 50 µg/mL dieckol treated cells showed increased red intensity fluorescence which clearly states the apoptotic induction of dieckol in A549 cell line (Figure 2).

The apoptotic induction of dieckol was confirmed by flow cytometry analysis using Annexin FITC stain and to further confirm the mitochondrial membrane potential disruption the cells were stained with JC‐1 stain. Compared with control there is increased number of early and late apoptotic cells in dieckol treated which is due to induction of apoptosis (Figures 3 and 4). Apoptosis are the programmed cell which is key target for most of the anticancer drugs. Caspases are proteases which majorly involved in innate immunity and it also plays s key role in regulating apoptosis.^30^ The caspases are classified into initiator caspases (caspase‐2, ‐8, ‐9 and 10) and executor caspases (caspase‐3, ‐6, ‐7).^31^ In the current study, dieckol increased the expression of both initiator caspases‐2,‐9 and the executor caspase‐3 (Figure 4), this may be the reason for increased apoptotic cells observed in the flow cytometric analysis of dieckol treated A549 cell. This results also correlates with the previous report were dieckol increased the expression of caspases‐2, ‐8, ‐9 in ovarian cancer SKOV3 cells.^32^

PI3K signaling plays a major role in cell survival, growth and proliferation.^33^ PI3K/AKT/mTOR signaling pathway is most commonly deregulated pathway in lung cancer.^34^ Most of the studies conducted on NSCLC revealed there is 50% to 70% increase in the expression of AKT protein due to the abnormal activation of PI3K/AKT/mTOR signaling.^35^ The drug which inhibits the over expression of PI3K/AKT/mTOR signaling molecules may be potent drug to treat lung cancer. Hence, we assessed the effect of dieckol on inhibiting the PI3K/AKT/mTOR signaling. PI3K are group of lipid kinases classified into three, among which class IA PI3K are most commonly deregulated in the cancer conditions.^36^ PI3K were activated by the receptor tyrosine kinases and the activated PI3K further activates AKT. Activated AKT inturn phosphorylates the downstream molecules PDK1 and mTOR, which on further activates the transcription factors responsible for the cell survival, growth and proliferation.^37^ AKT inhibitor GDC 0068 and mTOR inhibitor RAD‐001 are currently used to treat lung cancer patients in phase I trial,^38^ which has severe side effects. In the present study, dieckol a herbal based drug with nil side effects effectively inhibited the PI3K/AKT/mTOR signaling pathway and it also significantly decreased the expression of P70S6K and the transcription factor cyclin D1 which confirms dieckol as potent anticancer agent induces apoptosis via inhibiting PI3K/AKT/mTOR signaling pathway.

The invasion and migration are hallmark characters of cancer cells which depend on the external and internal signals such as adhesion receptor signaling, chemical signaling by chemokines and integrins.^39^ E‐cadherins are cell surface glucoproteins which plays a major role in epithelial to mesenchymal transition of cancer cells.^40^ Various studies reported the decrease in tumour suppressor protein E‐cadherin leads to cancer progression.^41^ The expression of E‐cadherin is regulated by various molecules like MAPK, Ras, and PI3K/AKT.^42^ Cadherin switch is an event which regulated by transcription factors such as TWIST, SNAIL, SLUG and so forth, leading to epithelial‐to‐mesenchymal transition (EMT).^43^ Kim et al^44^ reported pholoroglucinol effectively inhibited the genes N‐cadherin, SNAIL, TWIST, vimentin inducing EMT. In the present study also the expression of E‐cadherin is increased in dieckol treated whereas the expression of N‐cadherin, vimentin, TWIST, MMP‐9, and the urokinase plasminogen activator which is an extracellular matrix‐degrading protein were decreased (Figure 5). This may be the reason for the decrease in cell invasion and migration of dieckol treated A549 cell line during Transwell assay (Figure 5), which confirms the anticancer property of dieckol.

## 5 CONCLUSION

To conclude, lung cancer is the most prevalent cancer with lesser survival rate and treating it with potent drug causing nil or lesser side effects is the greatest challenge for the current clinicians. PI3K/AKT/mTOR signaling pathway plays a key role in cancer cell survival, proliferation and growth, hence, many research were focusing on the anticancer drug which specifically inhibits the PI3K signaling cascade. Dieckol is a one such potent anticancer drug which has inhibited the cell migration and invasion via inhibiting EMT signaling molecules and also in our present study it has induced apoptosis via inhibiting PI3K/AKT/mTOR signaling molecules. Hence, it can be subjected to future studies with clinical trials for treating lung cancer.
